RETRACTED

# Flat Panel CT Scanning Is Helpful in Predicting Hemorrhagic Transformation in Acute Ischemic Stroke Patients Undergoing Endovascular Thrombectomy

**DOI:** 10.1155/2021/5527101

**Published:** 2021-04-13

**Authors:** Liuwei Chen, Yi Xu, Rui Shen, Jiping Sun, Xiang Zhang, Quanbin Zhang, Feng Wang

**Affiliations:** ^1^Department of Neurosurgery, Shanghai Tenth People's Hospital, Tongji University School of Medicine, Shanghai, China; ^2^Departments of Neurology, Seventh People's Hospital of Shanghai University of Traditional Chinese Medicine, Shanghai, China

## Abstract

**Purpose:**

Hyperdense lesions are frequently revealed on flat panel CT (FP-CT) immediately after endovascular thrombectomy in patients with acute ischemic stroke. This study is aimed at discriminating hyperdense lesions caused by extravasation plus hemorrhage from those caused by contrast extravasation alone.

**Methods:**

We retrospectively analyzed clinical and radiological data of patients who underwent an immediate postprocedure FP-CT scan and a follow-up noncontrast CT 24 hours after thrombectomy. We especially focused on the Maximum Hounsfield Units (HU_max_) of each hyperdense lesion. A hyperdense lesion was judged to be hemorrhagic when it persisted on noncontrast CT and/or developed a mass effect.

**Results:**

Of 81 patients included in this study, 32 (39.5%) patients presented 41 hyperdense lesions on FP-CT. The chance of hemorrhagic transformation is higher in patients with hyperdense lesions on FP-CT than that in patients without hyperdense lesions (23/32 vs. 1/49, *p* < 0.001). The HU_max_ of hyperdensity on FP-CT can predict hemorrhagic transformation with an area under the curve of 0.805 (95% CI: 0.67-0.94, *p* = 0.02). The sensitivity, specificity, positive, and negative predictive values of hyperdensity on FP-CT for hemorrhagic transformation were 96%, 84%, 72%, and 98%, respectively. A HU_max_ of >600 predicted hemorrhagic transformation with a sensitivity of 50% and a specificity of 100%.

**Conclusions:**

The presence of hyperdensity on FP-CT can predict hemorrhagic transformation with a high sensitivity and negative predictive value. The measurement of HU_max_ of hyperdense lesion on FP-CT can be applied to the management of patients undergoing endovascular recanalization.

## 1. Introduction

Mechanical thrombectomy has been regarded as a milestone in the rescue of severe acute ischemic stroke (AIS) with high recanalization rates and dramatically improved results [1]. However, this endovascular treatment may result detrimental mainly because of hemorrhagic transformation (HT) [2]. Detection of intracerebral hemorrhage as early as possible is absolutely critical in the management of this intractable condition. Flat panel computed tomography (FP-CT) is a very useful tool for the detection of peri-interventional complications immediately after procedure without transferring patients to the CT unit [3, 4]. However, this imaging modality poses challenges in diagnosing HT in patients undergoing mechanical thrombectomy as the presence of hyperdense lesions could be either contrast extravasation alone or plus hemorrhage. The goal of this study was to evaluate the potential of FP-CT in the detection of intraparenchymal hemorrhage through analyzing Hounsfield Units of hyperdense areas seen on FP-CT immediately after mechanical thrombectomy.

RETRACTED

## 2. Methods and Materials

### 2.1. Patients

AIS patients who were treated with mechanical thrombectomy due to large vessel occlusion between January 2016 and March 2018 at our institution were retrospectively reviewed and analyzed. The inclusion criteria for the study were examined with an immediate postprocedure FP-CT and a follow-up noncontrast computed tomography (NC-CT) 24 hours after thrombectomy. Patients were excluded if their image data were incomplete or nondiagnostic due to motion or other artifacts. This study was approved by the ethics committee of our Institution, and the review board waived the need for written informed consent from the participants.

### 2.2. Stroke Management

In accordance with AHA/ASA guideline's acute ischemic stroke protocol, patients presenting large vessel occlusions within 6 hours from symptom onset received endovascular recanalization. A combination of Solitaire™ FR revascularization device and Navein guide catheter (ev3, Irvine, CA, USA) was employed for mechanical thrombectomy in all selected cases. Balloon or stent-assisted angioplasty as an alternative was performed only when stent retriever thrombectomy failed due to intracranial stenosis. Details on the arterial occlusion sites, median time from onset to puncture (onset-to-puncture time), procedure time, interval between FP-CT and NC-CT, and so on were recorded for each patient. Recanalization was considered to be successful when the thrombolysis in cerebral infarction (TICI) score was 2b or 3. Decompressive craniectomy was reserved for patients whose neurological condition deteriorated due to significant space-occupying effect. The neurologic outcomes were assessed using the modified Rankin scale (mRS) score at a three-month follow-up. Favorable outcomes were defined as scores ≤ 2.

### 2.3. Image Acquisition

FP-CT scans were regularly performed at the end of thrombectomy, while follow-up NC-CT scans were finished about 24 hours after the procedure. FP-CT scans were performed with a biplane angiography system (Dyna CT, Siemens, Germany) using the following parameters: voltage, 84 kV; tube current, 253 mA; acquisition time, 11.6 ms per frame; projection on 48 cm flat panel size; angulation, frame speed, 30 frames per second, 0.4° per frame; total angle, 196**°**; exposure time, 20 s. NC-CT images were acquired on a 64-slice multidetector CT (GE LightSpeed VCT, GE Healthcare, USA) at 120 kV, 250 mA, and 1.0 s rotation time. Images were reconstructed with 5 mm section thickness, using a standard reconstruction kernel, a field of view of 250 mm, and a 512 × 512 matrix.

RETRACTED

### 2.4. Image Analysis

Two experienced neurologists blinded to clinical data independently reviewed FP-CT images on a dedicated workstation (syngo Multi-Modality Workplace, Siemens, Germany) and NC-CT images on the PACS (Philips iSite PACS, Netherlands) in randomized order. Afterward, a consensus reading was performed to get a reference standard for statistical analyses.

Maximum Hounsfield Units (HU_max_) of hyperdense lesions in FP-CT were measured based on visually defined regions of interest. HU_max_ and location of each hyperdense lesion were separately recorded if there were multiple hyperdense lesions in the same patient. Hyperdense lesions that were no longer discernible on the follow-up NC-CT were regarded as contrast extravasation. Hyperdensity was confirmed to be hemorrhagic transformation (HT) when it persisted on NC-CT and/or developed a mass effect [5, 6]. HT was further categorized as symptomatic and nonsymptomatic. We defined symptomatic hemorrhage according to the SITS-MOST definition [7]: when blood clot exceeds 30% of the infarcted volume with significant mass effect or leads to a decline in NIHSS of ≥4 points or causing death within 36 hours.

### 2.5. Statistical Analysis

Continuous variables are expressed as the mean ± standard deviation, ordinal variables are expressed as median (interquartile), and categorical variables are expressed as numbers (frequencies). Bivariate comparisons were performed by the Mann–Whitney *U* test for continuous variables and the *χ*^2^ test for categorical variables (or Fisher's exact test when the expected cell frequency was <5). The sensitivity, specificity, positive predictive value, and negative predictive value of FP-CT for the prediction of HT were calculated. In addition, receiver operating characteristic analysis was performed to indicate the predictive value of the HU_max_ of hyperdensity for identifying intraparenchymal hemorrhage. All the statistical analyses were performed with SPSS version 21.0 (SPSS, Chicago, IL, USA). A value of *p* < 0.05 was considered to be significant.

## 3. Results

### 3.1. The Study Sample and Clinical Outcomes

Between January 2016 and March 2018, 87 patients underwent both FP-CT and follow-up NC-CT scans after mechanical thrombectomy but 6 were excluded due to poor image quality, yielding a cohort of 81 patients (49 males, 32 females). The mean age of this series was 67.4 ± 9.5 years (ranging from 49 to 83 years), and patients presented with a median on-admission NIHSS score of 15 (ranging from 6 to 26). The rate of successful recanalization (TICI 2b and 3) was 88.9% (72/81). Hyperdense lesions were found on 32 patients on the FP-CT. However, HT was revealed in 24 patients on the follow-up NC-CT, among them, 7 were symptomatic. At the 3-month follow-up, we obtained a functional independence rate of 45.7% (37/81) and a mortality rate of 11.1% (9/81). 6 patients died of symptomatic intracranial hemorrhage and/or brain infarction edema; the remaining 3 died because of systematic infection.

RETRACTED

According to the results of FP-CT scans, patients were divided into hyperdense lesion group (32 cases) and nonhyperdense lesion group (49 cases). There was no significant difference between the two groups regarding age, sex, occlusion sites, NIHSS scores, onset-to-puncture time, procedure time, interval between FP-CT and NC-CT, TICI scores, and so on (see Table 1); however, the rate of functional independence at 3 months was 53.1% (26/49) in the nonhyperdense lesion group and 34.3% (11/32) in the hyperdense lesion group (*p* = 0.12); meanwhile, the mortality rate is 6.1% (3/49) in the nonhyperdense lesion group, in comparison to 18.8% (6/32) in the hyperdense lesion group (*p* = 0.14), indicating that hyperdense lesion on FP-CT was related to unfavorable outcomes though statistical difference was not significant possibly due to sample size.

### 3.2. Hyperdensity Could Predict HT

The total number of HT was 24, most of them were from the hyperdense lesion group (23/32, 71.9%), and only one case was from the nonhyperdense lesion group (1/49, 2.0%). The difference was statistically significant (*p* < 0.001). The sensitivity and specificity of hyperdensity on FP-CT for detecting hemorrhage transformation were 96% (23/24) and 84% (48/57), respectively, while positive and negative predictive value were 72% (23/32) and 98% (48/49). Among the 24 cases with HT, 7 cases were categorized as symptomatic and all of them were from the hyperdense lesion group. Sample cases are shown in Figure 1.

There was a total of 41 hyperdense lesions in 32 patients, with 9 patients harboring two isolated hyperdense lesions. As 13 hyperdense lesions disappeared on the following NC-CT scans, they were attributed to oozing of contrast agent. The remaining 28 lesions were judged as hemorrhagic. The clinical features of these hyperdense lesions are shown in Table 2. We further divided the hyperdense lesions into the hemorrhagic group and the nonhemorrhagic group. The HU_max_ of each hyperdense lesion was measured, as a result, the HU_max_ of the hemorrhagic group was much higher than that of the nonhemorrhagic group (867.3 ± 667.1 verse 300.1 ± 127.0 HU, *p* = 0.02). It was very impressive that in one patient who had both hemorrhagic and nonhemorrhagic hyperdense lesions, the HU_max_ of the hemorrhagic one was much higher than that of the nonhemorrhagic one (Figure 2). The receiver operating characteristic analysis showed that the HU_max_ of the hyperdensity on FP-CT can predict HT with an area under the curve of 0.805 (95% CI: 0.67-0.94, *p* = 0.02) (Figure 3). The lowest and highest HU_max_ was 169 and 2766, respectively, in the 41 hyperdense lesions. With the upregulation of the threshold values, the sensitivity of HU_max_ for detecting HT decreased, but the specificity increased meanwhile. The highest HU_max_ of hyperdense lesion finally judged to be contrast extravasation was 561 HU, so when we set HU_max_ 600 by Youden index as a threshold value, it can predict HT with a sensitivity of 50% (14/28) and a specificity of 100%.

RETRACTED

## 4. Discussion

FP-CT has the advantage of immediately revealing peri-procedural abnormal conditions without transferring patients, which is especially useful in the management of patients undergoing endovascular recanalization.

Our study found that 39.5% of patients (32/81) had hyperdense lesions after mechanical thrombectomy, which is in line with previous reports (from 30% to 87% using NC-CT [8–15] and 16% to 60% using FP-CT [16–18]). As HT is critical in the setting of therapy for AIS patients, we attempted to investigate the potential of FP-CT in the prediction of HT. As a result, the hyperdense lesion on FP-CT demonstrated high sensitivity and negative predictive value for the detection of HT. When focusing on the HU_max_ of hyperdense lesions, we found that, with the increase of the HU_max_ value, the risk of HT enhanced accordingly. Berger et al. [19] reported that symptomatic intracranial hemorrhage was the only HT that independently caused clinical deterioration and impacted prognosis. As far as symptomatic hemorrhage is concerned, all the symptomatic cases are from the FP-CT (+) group, indicating that FP-CT can reliably predict symptomatic intracranial hemorrhage.

As a dynamic interface between the peripheral circulation and the central nervous system, the blood-brain barrier (BBB) controls the influx and efflux of biological substances needed for the brain metabolic processes, as well as for neuronal function. In the case of acute ischemic stroke, the damage to the BBB is initiated immediately after arterial occlusion, and the extent of BBB disruption is associated with the type, severity, and duration of ischemic insults. When the BBB disruption is relatively mild, the contrast agent is allowed to extravasate due to the increased permeability; however, with the progression of the ischemic/reperfusion injuries, the rupture of the blood-brain barrier takes place, leading to a massive extravasation of both contrast agent and blood elements [20]. Therefore, it is not difficult to explain why patients with hyperdense lesions on FP-CT have more chance of HT than those without hyperdense lesions, and the higher the HU_max_ of the hyperdense lesions, the greater the risk of symptomatic intracranial hemorrhage.

RETRACTED

The measurement of HU_max_ of the hyperdense lesions on FP-CT can be applied to the management of patients receiving endovascular recanalization. A large amount of data suggests that intracranial hemorrhage tends to occur within the first 12–24 hours after treatment [21]. It is proper to delay antiplatelet and anticoagulant drugs when a hyperdense lesion is found on FP-CT until a follow-up NC-CT is performed to rule out hemorrhage. Blood pressure management is another urgent consideration in these patients. Target blood pressure is set according to the recanalization level of the occluded circulation. A systolic blood pressure goal of less than 140 mmHg is recommended for those achieving successful recanalization [22]; however, if hyperdense lesions are presented, neurocritical care, including sedation, analgesia, and strict blood pressure control, is recommended to reduce the risk of HT. When HU_max_ of the hyperdense lesion breaks a threshold value (600 HU in our study), hemorrhage is almost inevitable, preparation for decompressive craniectomy in advance is strongly suggested when extensive hyperdense lesions are found on FP-CT, considering that the final infarction area can be evaluated on the basis of hyperdense lesions [23].

Recanalization of the responsible cerebral vessels is the primary target after the onset of AIS; however, the big gap between the high recanalization rate and the relatively low functional independence rate implies the revascularization in a large proportion of patients is actually futile or even detrimental. How to select the best candidates for recanalization is still a hot topic at present. As FP-CT has the advantage of providing real-time information on the integrity of the blood-brain barrier, the final decision to restore or not to restore the blood flow could be made by referring to the FP-CT image, especially in a dilemma moment. Takes it for example, after temporary blood flow restoration with the deployment of a stent retriever, we can perform an FP-CT scan, if extensive hyperdense lesions already exist while stenting and antiplatelet administration are necessary to achieve a successful recanalization. It is sagacious to abandon recanalization, as the risk of symptomatic hemorrhage is very high after reperfusion.

RETRACTED

## 5. Limitations

Our study has several limitations. First, our study was performed retrospectively with a small sample size from a single center, which might result in selection bias. In addition, the amount of contrast media and the number of recanalization attempts were reported to be risk factors for HT [24, 25]; in our study, the dose, volume, type of contrast media administered, and number of recanalization attempts were not available in some patients, which made the evaluation limited.

## 6. Conclusions

The presence of hyperdensity on FP-CT can predict HT with a high sensitivity and negative predictive value. The measurement of HU_max_ of hyperdense lesion on FP-CT can be applied to the management of patients undergoing endovascular recanalization.

## Figures and Tables

**Figure 1:** Images of sample patients. A 56-year-old man with acute occlusion of the left middle cerebral artery (a) received successful recanalization (b). Flat panel CT shows hyperdense lesion in the head of the left caudal nucleus (c), which resolved on noncontrast CT 24 hours after thrombectomy (d). A 67-year-old man with acute occlusion of the right internal carotid artery (e) received successful recanalization (f). Flat panel CT shows hyperdense lesion in the right basal ganglia and right middle cerebral artery territory (g), which persisted on noncontrast CT (h).

**Figure 2:** Images of post-procedure flat-panel CT (a) and non-contrast CT (b) in one patient. Flat panel CT shows hyperdensity in the left basal ganglia and left temporosphenoid lobe. The HU_max_ of left basal ganglia is 1405 and the HU_max_ of left temporosphenoid lobe is 474. Noncontrast CT revealed hemorrhage only in the left basal ganglia.

**Figure 3:** Receiver operating characteristic curve for the predictive value of HU_max_ for hemorrhagic transformation. The HU_max_ value was a predictor of hemorrhagic transformation with statistical significance (area under curve of 0.805; 95% CI: 0.67-0.94, *p* = 0.02).

**Table 1:** Comparisons of hyperdensity versus no hyperdensity on flat panel CT performed immediately after mechanical thrombectomy.

	FP-CT+ (*N* = 32)	FP-CT- (*N* = 49)	*p*
HT	23 (71.9%)	1 (2.0%)	*p* < 0.01
Age in years	66.2 ± 10.9	66.9 ± 8.6	0.45
Male	19 (59.4%)	30 (61.2%)	>0.99
Baseline NIHSS score	15 (13-18)	15 (12-18)	0.54
Occluded circulation			0.85
Anterior	26 (81.2%)	39 (79.6%)	
Posterior	6 (18.8%)	10 (20.4%)	
Occluded arteries			0.98
MCA isolated	18 (56.2%)	27 (55.1%)	
ICA isolated or tandem with MCA	8 (25.0%)	12 (24.5%)	
Posterior circulation	6 (18.8%)	10 (20.4%)	
Time from symptom onset to puncture	210.2 ± 64.8	195.7 ± 80.9	0.15
Procedure time	103.0 ± 44.1	91.1 ± 32.2	0.24
Interval between FP-CT and NC-CT	25.1 ± 3.9	23.7 ± 3.5	0.37
Recanalization after treatment,			0.25
TICI < 2b	5 (15.6%)	3 (6.1%)	
TICI ≥ 2b	27 (84.4%)	46 (93.9%)	
3-month mRS			0.12
≤2	11 (34.4%)	26 (53.1%)	
>2	21 (65.6%)	23 (46.9%)	
Mortality rate	6 (18.8%)	3 (6.1%)	0.14

Data are *n* (%), median (interquartile), or mean ± standard deviation. Note: FP-CT indicates flat panel CT, HT indicates hemorrhagic transformation, NIHSS indicates National Institutes of Health Stroke Scale, MCA indicates middle cerebral artery, ICA indicates internal carotid artery, TICI indicates thrombolysis in cerebral infarction, mRS indicates modified Rankin scale.

RETRACTED

**Table 2:** The clinical features of patients with hyperdense lesions on FP-CT.

Variable	Total hyperdense lesions (*n* = 41)	Hemorrhagic lesions		*p*
		Yes (*n* = 28)	No (*n* = 13)	
Age	68.6 ± 11.2	67.5 ± 11.4	70.9 ± 10.8	0.34
Sex (male)	25 (61.0%)	19 (67.9%)	6 (46.2%)	0.18
Baseline NIHSS score	15 (12-18)	16 (13-20)	14 (11-14)	0.08
Occluded arteries (*n*, %)				0.05
MCA isolated	21 (51.2%)	11 (39.3%)	10 (76.9%)	
ICA isolated or tandem with MCA	14 (34.1%)	11 (39.3%)	3 (23.1%)	
Posterior circulation	6 (14.6%)	6 (21.4%)	0 (0.0%)	
Time from symptom onset to puncture	204.8 ± 66.3	211.9 ± 65.9	189.6 ± 67.4	0.31
Procedure time	105.1 ± 42.7	109.0 ± 45.8	96.5 ± 35.0	0.58
Interval between FP-CT and NC-CT	25.0 ± 4.1	24.5 ± 4.1	26.0 ± 4.1	0.20
Recanalization after treatment				0.39
TICI < 2b	6 (14.6%)	5 (17.9%)	1 (7.7%)	
TICI ≥ 2b	35 (85.4%)	23 (82.1%)	12 (92.3%)	
3-month mRS				0.55
≤2	12 (29.3%)	9 (32.1%)	3 (23.1%)	
>2	29 (70.7%)	19 (67.9%)	10 (76.9%)	
Mortality rate	8 (19.5%)	8 (28.6%)	0 (0.0%)	0.03
HU_max_	687.4 ± 613.7	867.3 ± 667.1	300.1 ± 127.0	0.02

Data are *n* (%), median (interquartile), or mean ± standard deviation. Note: HU_max_ indicates maximum Hounsfield units.

## Data Availability

The data used to support the findings of this study are available from the corresponding author upon request.
